The article "Role of short-wavelength blue light in the formation of cataracts and the expression of caspase-1, caspase-11, Gasdermin D in rat lens epithelial cells: insights into a novel pathogenic mmechanism of cataracts" was retracted in 2022. Reasons: errors in the data; concerns about the data; concerns about the images; concerns about the results or conclusions.

# Role of short-wavelength blue light in the formation of cataracts and the expression of caspase-1, caspase-11, Gasdermin D in rat lens epithelial cells: insights into a novel pathogenic mmechanism of cataracts

**DOI:** 10.1186/s12886-020-01565-z

**Published:** 2020-07-15

**Authors:** Yamin Wang, Min Zhang, Ying Sun, Xiaohui Wang, Zhaowei Song, Huazhang Li, Kexin Liu, Zhijian Li

**Affiliations:** 1 Department of Ophthalmology, the First Affiliated Hospital, Harbin Medical University, 143 Yiman Street, Nangang District, Harbin, China; 2 Department of Ophthalmology, the 2nd Hospital of Heilongjiang, Harbin, China

**Keywords:** Pyroptosis, Short-wavelength blue light, Caspase-1/11, GSDMD, Cataract

## Abstract

**Background:**

With the popularity of blue-rich light-emitting diode (LED)-backlit display devices, our eyes are now exposed to more short-wavelength blue light than they were in the past. The goal of this study was to investigate the pathogenesis of cataracts after short-wavelength light exposure.

**Methods:**

Sprague-Dawley (SD) rats were selected and randomly divided into a control group (10 rats each for the 4-, 8-, and 12-week groups) and an experimental group (10 rats each for the 4-, 8-, and 12-week groups). The rats in the experimental group were exposed to a short-wavelength blue LED lamp for 12 h per day. After exposure to the blue LED lamp, the rats were maintained in total darkness for 12 h, after which a 12-h light/dark cycle was resumed. The intensity of the lamp was 3000 lx. At the end of the short-wavelength blue LED lamp exposure (for 4, 8, and 12 weeks), the expression levels of caspase-1, caspase-11 and gasdermin D (GSDMD) were examined in rat lens epithelial cells (LECs) using qRT-PCR and Western blot analyses. An illuminance of 2500 lx was used to study the potential effect of blue LED light on HLE-B3 hLECs in vitro**.** AC-YVAD-CMK, a caspase-1 inhibitor, was used to confirm the pyroptosis of LECs by flow cytometry.

**Results:**

After 6 weeks, cataracts developed in the experimental rats (4/20 eyes). The clarity of the lens gradually worsened with the duration of exposure. Twelve weeks later, all of the rat eyes had developed cataracts. The expression levels of caspase-1, caspase-11 and GSDMD at 4, 8, and 12 weeks were significantly higher in the samples from rats exposed to a short-wavelength blue LED lamp than in the samples from control rats (*p*<0.05). The proportions of double-positive hLECs were significantly increased in the 5-h and 10-h short-wavelength blue light exposure subgroups compared with the 5-h and 10-h caspase-1 inhibitor subgroups (*p* < 0.05).

**Conclusion:**

The data indicate that pyroptosis plays a key role in cataract induction after short-wavelength blue light exposure. This study might provide new insights into a novel pathogenic mechanism of cataracts.

The article "Role of short-wavelength blue light in the formation of cataracts and the expression of caspase-1, caspase-11, Gasdermin D in rat lens epithelial cells: insights into a novel pathogenic mmechanism of cataracts" was retracted in 2022. Reasons: errors in the data; concerns about the data; concerns about the images; concerns about the results or conclusions.

## Background

Globally, cataracts are the leading cause of blindness and account for nearly half (47.8%) of all blindness cases [1, 2]. In a study in rural northern China, approximately 28.6% of participants aged 50 and older had poor postoperative visual outcomes, and cost was the most common barrier (73.9%) to cataract removal [3]. To date, the only effective therapeutic method for cataracts is surgery, which has the potential for serious postoperative complications, e.g., increased intraocular pressure (IOP) and corneal edema. Hence, studies of cataractogenesis are vital for developing effective therapeutic modalities for the prevention and treatment of cataracts.

Cataracts are associated with a number of risk factors, e.g., drugs, malnutrition, aging, exposure to ultraviolet (UV) light, and diabetes mellitus [4–6]. Short-wavelength blue light (400–500 nm) has attracted increasing attention because of its potential to injury the retina [7, 8]. The relationship between the formation of cataracts and short-wavelength blue light exposure has been mentioned, but the evidence is inconclusive.

Apoptosis and pyroptosis rely on specific caspases to induce their respective programmed cell death pathways [9]. Inflammatory caspases (caspases-1, − 4, − 5 and − 11) induce a form of necrotic programmed cell death, namely, pyroptosis, which is motivated by the canonical and noncanonical inflammasome signaling pathways [10–14]. The activity of caspase-1 leads to the maturation of IL-1β and IL-18 and the cleavage of gasdermin D (GSDMD) to induce pore opening [15–17]. Accumulating evidence has confirmed that pyroptosis is involved in the pathogenesis of both noninfectious and infectious diseases [18, 19].

In the present study, we hypothesized that pyroptosis is involved in the pathogenesis associated with the occurrence and development of cataracts. A rat model of short-wavelength blue light exposure was established, and relative changes in pyroptosis factors in rat lens epithelial cells (LECs) were analyzed.

## Methods

### Animals

Six-week-old male SD rats (weighing 210 ± 30 g) were provided by the Central Laboratory of the First Affiliated Hospital of Harbin Medical University, China. The housing conditions were as follows: room temperature (18–25 °C), 75% humidity, and 10 rats per cage. This study was carried out according to the GCULA of the NIH. The study protocol was approved by the Ethics Committee of the First Affiliated Hospital, Harbin Medical University, China.

SD rats were selected and randomly divided into a control group (10 rats each for the 4-, 8-, and 12-week groups) and an experimental group (10 rats each for the 4-, 8-, and 12-week groups). The rats in the control group were exposed to continuous indoor natural light from 6 AM to 6 PM and were then maintained on a daily routine of total darkness (12 h indoor natural light/dark cycle). The light exposure experiment in the rat model was carried out in Harbin, China (44°04′-46°40′N) from July 2018 until September 2018. The average intensity of indoor natural light showed a maximum of 2100 lx around noon.

The article "Role of short-wavelength blue light in the formation of cataracts and the expression of caspase-1, caspase-11, Gasdermin D in rat lens epithelial cells: insights into a novel pathogenic mmechanism of cataracts" was retracted in 2022. Reasons: errors in the data; concerns about the data; concerns about the images; concerns about the results or conclusions.

The rats in the experimental group were exposed to a short-wavelength blue light-emitting diode lamp (455–460 nm) (Grass Farmer’s Home Co., Ltd., Shenzheng, China) as previously described [20]. The rats were maintained in a 12-h blue light/dark cycle. An illuminance of 1000–3000 lx was selected to investigate the roles of light in retinal injury in previous studies [21–23]. In the present research, we adopted an illuminance intensity of 3000 lx to study the potential influence of blue light on rat lenses. All rats in both groups were treated with atropine gel to induce mydriasis.

At the end of exposure to a short-wavelength blue LED lamp (4, 8, and 12 weeks), the lens clarity changes in all rats were examined, and the rats in each group were sacrificed by cervical dislocation under anesthesia as described previously [24]. Both eyes were rapidly enucleated, and the intact lenses were removed after the rats were confirmed dead. The lens capsules from both eyes were used for one experiment.

### Cell culture

The HLE-B3 hLEC line (provided by ATCC, Manassas, VA, USA) was cultured as a monolayer in DMEM as previously described [25]. The cells were inoculated onto 6-well plates (5 × 10^5^–1 × 10^6^ cells) for the experiments as described previously [23]. The protective effects of AC-YVAD-CMK against short-wavelength blue light were investigated. The concentration of AC-YVAD-CMK was determined by a CCK-8 assay (SAB, USA) [26]. The HLE-B3 LECs were grouped into 3 groups as follows: A: the control group, which consisted of hLECs cultured in the dark; B: the caspase-1 inhibitor group, which consisted of HLE-B3 hLECs treated with AC-YVAD-cmk (20 μmol/L); and C: the short-wavelength blue light exposure group. Groups B and C were subdivided into four subgroups according to the blue light exposure time (5 h and 10 h).

### Short-wavelength blue light exposure

Experimental illumination systems (455–460 nm) were installed on top of the cell culture incubator as previously described. We adopted an illuminance of 2500 lx [26] to study the potential influence of blue LED light on hLECs.

The article "Role of short-wavelength blue light in the formation of cataracts and the expression of caspase-1, caspase-11, Gasdermin D in rat lens epithelial cells: insights into a novel pathogenic mmechanism of cataracts" was retracted in 2022. Reasons: errors in the data; concerns about the data; concerns about the images; concerns about the results or conclusions.

### Flow cytometry

A cell viability assay of LECs was performed via flow cytometry in 6-well plates [27]. When pyroptosis occurs in cells, membrane permeability increases. PI can enter the cells and stain the DNA, while phosphatidylserine (PS) is on the inside of the cell membrane and can be stained by an antibody (Annexin V). Therefore, flow cytometry was used to distinguish pyroptosis from apoptosis, and double-positive staining of PI and Annexin V occurs in cell pyroptosis [28].

### Quantitative real-time PCR (qRT-PCR)

qRT-PCR was used to examine the relative expression of caspase-1, caspase-11, and GSDMD in all control and experimental rat LEC samples as previously described [23]. Five SD rats were used for each experimental time point in qRT-PCR.

### Western blot analysis

Western blotting was performed to quantify tissue protein expression as previously described [23]. Detailed methods and tables are provided in the supplementary materials. Five SD rats were used for each experimental time point in Western blotting.

### Statistical analyses

Statistical analyses were performed using SPSS 23.0 software (SPSS Inc., USA). Data are given as the mean ± standard deviation (SD). Differences between groups were analyzed by two-way ANOVA. *p* < 0.05 was considered significant.

## Results

### Effects of short-wavelength blue light on cataract formation

The lenses of the rats in the control group appeared transparent throughout the 12-week observation period. At 4 weeks after short-wavelength blue LED lamp exposure, all rat lenses in both the control and experimental groups were transparent (Fig. 1). However, after 6 weeks, cataracts had developed in the experimental rats (4/20 eyes), as indicated by equatorial and postcortical vacuoles (grade 2). After 8 weeks of exposure, 25% (5/20 eyes) of the rat eyes displayed grade 2 cataracts, and 25% (5/20 eyes) displayed grade 3 cataracts (Fig. 1). Twelve weeks later, 100% of the rat eyes exposed to blue light exhibited cataracts. Of all the eyes with cataracts, 55% (11/20 eyes) of the rat eyes displayed grade 2 cataracts, 25% (5/20 eyes) displayed grade 3 cataracts, and 20% (4/20 eyes) displayed mature cataracts (grade 4) (Fig. 1).

**Fig. 1:** Slit-lamp observation images of rat lenses. **a**: Control group: the rat lenses were all transparent. **b**: Experimental group: grade 2 cataract. **c**: Experimental group: grade 3 cataract. **d**: Experimental group: grade 4 cataract

### Morphologic changes in HLE-B3 hLECs

The dynamic morphologic changes of HLE-B3 hLECs under short-wavelength blue light exposure were observed under an inverted microscope in the culture room (Fig. 2). The cells in the control group were uniformly distributed, and the cell membrane was intact. After 5 h of short-wavelength blue light exposure, the morphological changes of the cells were not obvious, and the cell distribution was relatively uniform. However, after 10 h of exposure, the number of cells in group C was decreased significantly, and the cell morphology appeared slightly swollen. The results indicated that short-wavelength blue light can cause cell death in HLE-B3 hLECs in a time dependence manner.

The article "Role of short-wavelength blue light in the formation of cataracts and the expression of caspase-1, caspase-11, Gasdermin D in rat lens epithelial cells: insights into a novel pathogenic mmechanism of cataracts" was retracted in 2022. Reasons: errors in the data; concerns about the data; concerns about the images; concerns about the results or conclusions.

**Fig. 2:** Morphological changes of hLECs under short-wavelength blue light exposure (400×). **a** Control group: morphology change of the HLE-B3 hLECs in the non-light culture. The cell membrane was intact. **b** After 5 h of short-wavelength blue light exposure, the morphological changes of the cells were not obvious. **c** After 10 h of blue light exposure, the number of cells was decreased significantly, and the cells appeared slightly swollen

### Short-wavelength blue light can cause pyroptotic cell death

Pyroptotic programmed cell death was evaluated according to double-positive staining using flow cytometry. In the caspase-1 inhibitor group, the proportions of double-positive hLECs were increased in the 5-h and 10-h subgroups compared with the control group (*p* < 0.05) (Fig. 3). The proportion of double-positive hLECs increased in a time dependence manner. In the short-wavelength blue light group, the proportion of double-positive hLECs also showed the same trend. Moreover, the proportions of double-positive hLECs were significantly increased in the 5-h and 10-h short-wavelength blue light exposure subgroups compared with the 5-h and 10-h caspase-1 inhibitor subgroups (*p* < 0.05).

**Fig. 3:** Double-positive staining for caspase-1 was performed using flow cytometry. **a**. Representative images of double-positive staining evaluated using flow cytometry. **b**. Proportions of double-positive cells. Group B: caspase-1 inhibitor group; Group C: short-wavelength blue light group; and NC: normal control group. The proportions of double-positive hLECs were significantly increased in the 5-h and 10-h subgroups in both groups B and C. *n* = 5. ^*^p < 0.05

### Expression of caspase-1

To determine whether caspase-1 was associated with changes in rat eyes after exposure to a short-wavelength blue LED lamp, we examined the relative expression of caspase-1 in all control and experimental rat LEC samples using qRT-PCR. The relative expression levels of caspase-1 were significantly higher in samples from short-wavelength blue LED lamp-exposed rats at 4, 8, and 12 weeks than in those from control rats at the corresponding time points (*p*<0.01) (Fig. 4). This study also showed that caspase-1 expression levels were higher in the 12-week group than in the 4-week and 8-week blue light exposure groups.

The article "Role of short-wavelength blue light in the formation of cataracts and the expression of caspase-1, caspase-11, Gasdermin D in rat lens epithelial cells: insights into a novel pathogenic mmechanism of cataracts" was retracted in 2022. Reasons: errors in the data; concerns about the data; concerns about the images; concerns about the results or conclusions.

**Fig. 4:** The relative expression of caspase-1 using qRT-PCR. The values of the control group were considered to be 1. The expression levels of caspase-1 in the blue light exposure group (4, 8, and 12 weeks) were increased compared with those in the control group (**p < 0.01). However, no significant difference was established with the control group at 4, 8 and 12 weeks (*p* > 0.05)

Western blot analysis revealed that caspase-1 protein expression was upregulated in the experimental group (4, 8 and 12 weeks after short-wavelength blue light exposure) compared to the control group at the same time points (*p* < 0.05) (Fig. 5). The present results indicate that short-wavelength blue LED lamp exposure is associated with increased expression of caspase-1 in rat LECs.

**Fig. 5:** The expression of cleaved caspase-1 in rat LECs using Western blot. Significant differences were not observed between the blue light exposure group and the control group at 4 weeks (*p* = 0.057). The expression levels of caspase-1 in the blue light exposure group (8- and 12-week groups) were increased compared with those in the control group (*p < 0.05)

### Expression of caspase-11

We investigated the mRNA expression levels of caspase-11. Caspase-11 mRNA expression was significantly higher in rats exposed to short-wavelength blue light (4-, 8-, and 12-week blue light exposure groups) than in healthy control rats (*p* < 0.05). Caspase-11 expression levels in the 8-week and 12-week blue light exposure group samples were increased compared to those in the 4-week blue light exposure group (*p* < 0.05) (Fig. 6). These results revealed that short-wavelength blue light exposure could induce pyroptosis in rat lens cells in a time dependence manner.

**Fig. 6:** The relative expression of caspase-11 using qRT-PCR. The values of the control group were considered to be 1. The expression levels of caspase 11 in the blue light exposure group (4, 8, and 12 weeks) were increased compared with those in the control group. (*p < 0.05, **p < 0.01)

As shown in Fig. 7, compared with the control group, the experimental groups exhibited markedly increased protein expression of cleaved caspase-11 in rat LECs at 4, 8 and 12 weeks. Furthermore, the cleaved caspase-11 levels were also higher in rat lens cells after 12 weeks of short-wavelength blue light exposure than in rat lens cells after 4 and 8 weeks of exposure (*p* < 0.05).

**Fig. 7:** The relative expression of cleaved caspase-11 using Western blot. The expression levels of cleaved caspase-11 in the blue light exposure group (4, 8, and 12 weeks) were increased compared with those in the control group (*p < 0.05). However, significant differences from the control group were not established (*p* > 0.05)

The article "Role of short-wavelength blue light in the formation of cataracts and the expression of caspase-1, caspase-11, Gasdermin D in rat lens epithelial cells: insights into a novel pathogenic mmechanism of cataracts" was retracted in 2022. Reasons: errors in the data; concerns about the data; concerns about the images; concerns about the results or conclusions.

### Expression of GSDMD

The GSDMD activity in rat lens cells subjected to short-wavelength blue light exposure was also measured using qRT-PCR in this study (Fig. 8). GSDMD expression was significantly increased after 4, 8 and 12 weeks of short-wavelength blue light exposure, and longer exposure times at the same intensity had more dramatic effects on the increase in GSDMD expression (*p* < 0.05).

**Fig. 8:** The expression of GSDMD using qRT-PCR. The values of the control group were considered to be 1. The expression levels of GSDMD in the blue light exposure group (4, 8, and 12 weeks) were increased compared with those in the control group (*p < 0.05, **p < 0.01), and the expression of GSDMD in the experimental group increased gradually with time

In the present study, Western blot analysis using an anti-GSDMD antibody was performed to investigate the change in GSDMD expression levels in rat LECs after 4, 8, and 12 weeks of short-wavelength blue light exposure. Cleaved GSDMD levels increased after short-wavelength blue light exposure, and as the exposure time increased, cleaved GSDMD expression increased (Fig. 9).

**Fig. 9:** The relative expression of GSDMD using Western blot. The expression levels of cleaved GSDMD in the blue light exposure group (4, 8, and 12 weeks) were increased compared with those in the control group (*p < 0.05), and the expression levels of cleaved GSDMD in the experimental group increased with time. However, significant differences from the control group were not established (*p* > 0.05)

## Discussion

LED light will gradually replace traditional incandescent light due to its considerable advantages, such as low power consumption and high light efficiency. However, the possible bio-photochemical injury to the eyes caused by LED light has also aroused public concern [29]. Previous studies have shown that blue light induced oxidative stress and cellular damage in retinal tissues [30–32]. In agreement with these findings, blue light-filtering IOLs have been thought to be a protective measure against blue light damage to the retina [33]. Studies have confirmed that cumulative visible light exposure may accelerate the development of cataracts [34]. Dysfunction of the LECs may lead to superficial cortical lens fiber edema and mature cataracts [35].

An increasing number of studies have focused on elucidating the mechanisms of pyroptosis in different diseases. In our study, we report that after 6 weeks of short-wavelength blue LED lamp exposure, cataracts developed in the experimental rats. In addition, pyroptosis markers, including caspase-1, caspase-11, and GSDMD, were investigated. The present study showed that the expression levels of caspase-1, caspase-11 and GSDMD were significantly increased in rat LECs after 4, 8, and 12 weeks of exposure to a short-wavelength blue LED lamp. The results confirmed that pyroptosis may play a vital role in the formation of cataracts after short-wavelength blue light exposure.

The article "Role of short-wavelength blue light in the formation of cataracts and the expression of caspase-1, caspase-11, Gasdermin D in rat lens epithelial cells: insights into a novel pathogenic mmechanism of cataracts" was retracted in 2022. Reasons: errors in the data; concerns about the data; concerns about the images; concerns about the results or conclusions.

Our present research demonstrated that cataracts had developed in the experimental rats after 6 weeks of blue light exposure. The clarity of the lens then progressively worsened with the duration of short-wavelength blue light exposure. The process of cataract formation illustrated in this study is consistent with that reported in an earlier study [35]. In this study, the phenotype is a cataract involving lens fiber cells. The cell culture results also indicated that short-wavelength blue light can cause cell death in HLE-B3 hLECs with time.

A previous study demonstrated that pyroptosis participates in the oxidation of human LECs and may be involved in the initiation and progression of noncongenital cataracts. Caspase-1 plays an important role in the process of pyroptosis during the formation of cataracts [36]. However, the role of short-wavelength blue light in the cataracts formation and the relative expression of pyroptosis markers, such as caspase-1, caspase-11, and GSDMD, in vivo is still unknown. In the present study, we demonstrated that short-wavelength blue light-induced activation of caspase-1, caspase-11, and GSDMD triggered cataracts in a pyroptosis-dependent manner.

Caspase-1, which is a crucial marker of the process of pyroptosis [37], is activated by the NLRP3 inflammasome. Caspase-1 mediates proinflammatory programmed cell death in response to exogenous and endogenous stimuli to protect cells. The results of the current study show that caspase-1 expression levels were increased in short-wavelength blue light-exposed rat lens cells in a dose-dependent manner.

Most previous studies have focused on targeting the canonical inflammasome pathway. However, emerging studies have actively explored the regulatory role of the noncanonical caspase-11 inflammasome in noninfectious diseases. Studies have indicated that aging activates the NLRP1 inflammasome, resulting in the processing of caspase-1 and the upregulation of caspase-11 [38]. Assembly and activation of the NLRP1 inflammasome involves caspase-1 and caspase-11 activation, which subsequently leads to the maturation and secretion of IL-1β and IL-18 [39, 40]. In the present study, the qRT-PCR and Western blot analysis results showed increased expression of caspase-11 in rat LECs after short-wavelength blue light exposure. We hypothesize that caspase-11 might be activated by naturally occurring intracellular molecules under inflammatory conditions and that these intracellular inflammatory molecules might bind directly to caspase-11, subsequently activating caspase-11 noncanonical inflammasomes and leading to the pathogenesis of cataracts after short-wavelength blue light exposure. Further investigation is required to confirm this hypothesis.

The article "Role of short-wavelength blue light in the formation of cataracts and the expression of caspase-1, caspase-11, Gasdermin D in rat lens epithelial cells: insights into a novel pathogenic mmechanism of cataracts" was retracted in 2022. Reasons: errors in the data; concerns about the data; concerns about the images; concerns about the results or conclusions.

Studies have revealed that GSDMD is activated by caspases − 1, − 4, − 5, and − 11, all of which split GSDMD into an N-terminal effector domain and a C-terminal inhibitory domain [17, 41]. We found that the mRNA expression levels of GSDMD were increased, suggesting that pyroptosis was activated by short-wavelength blue light. Additional morphological evidence of gasdermin-mediated pore formation and membrane rupture in LEC pyroptosis is also needed.

Furthermore, we used annexin V-FITC/PI together with flow cytometry to analyze the percentage of viable cells and the pyroptosis of HLE-B3 cells after short-wavelength blue light exposure for different times. The evaluation method was a strength of this work. Our results suggested that short-wavelength blue light exposure caused pyroptotic death in HLE-B3 hLECs with time. As expected, the caspase-1 inhibitor may effectively suppress the formation of cataracts and defend against LEC damage by suppressing the caspase-1/GSDMD pathway under short-wavelength blue light exposure.

Our study has potential limitations. The increased levels of caspases and GSDMD in SD rats, which are nocturnal, and in the albino strain, do not thoroughly explain the association between short-wavelength blue light exposure and the formation of cataracts in humans. Other inflammatory responses in the cornea, conjunctiva, and anterior chamber must be investigated to understand the precise mechanism of cataract formation under short-wavelength blue light exposure. Second, the intensity and duration of the blue light used in the study were not physiologically relevant, and additional studies on the safety of long-term exposure to low levels of blue light are needed to determine the effects of blue light on the eye. Finally, although the increased level of caspase-1 may suggest that pyroptosis is involved in this process, it is difficult to determine whether other cell death types, such as apoptosis and necrosis, are concurrently involved in cataract formation in lens cells exposed to short-wavelength blue light. Therefore, further research is needed to address this issue. We will also focus on studying the pathogenesis of cataracts under short-wavelength blue light in vitro, and ROS changes will be included.

The article "Role of short-wavelength blue light in the formation of cataracts and the expression of caspase-1, caspase-11, Gasdermin D in rat lens epithelial cells: insights into a novel pathogenic mmechanism of cataracts" was retracted in 2022. Reasons: errors in the data; concerns about the data; concerns about the images; concerns about the results or conclusions.

## Conclusions

We demonstrated that the expression of the pyroptosis markers caspase-1, caspase-11, and GSDMD in rat LECs was increased after short-wavelength blue light exposure. Thus, therapeutic strategies that aim to prevent LEC pyroptosis may inhibit the expression of related pyroptotic factors and may be beneficial for treating age-related cataracts.

## Supplementary information

**Additional file 1.**

## Data Availability

The datasets used during this current study are available from the corresponding author on reasonable request.

## Abbreviations

LED: Light-emitting diode
LECs: Lens epithelial cells
IOP: Intraocular pressure
UV: Ultraviolet light
GSDMD: Gasdermin D
NLRs: NOD-like receptors
GCULA: Guide for the Care and Use of Laboratory Animals
NIH: National Institutes of Health
ATCC: American Type Culture Collection
CCK-8: Cell counting kit-8
LPS: Lipopolysaccharide
GAPDH: Glyceraldehyde 3-phosphate dehydrogenase
PBS: Phosphate-buffered saline
IOLs: Intraocular lenses
hLECs: Human lens epithelial cells
